This article has been retracted.

# Downregulation of *SUMO2* inhibits hepatocellular carcinoma cell proliferation, migration and invasion

**DOI:** 10.1002/2211-5463.13173

**Published:** 2021-05-14

**Authors:** Jintu Chen, Canwei Chen, Yongfa Lin, Yongfa Su, Xueping Yu, Yancheng Jiang, Zixuan Chen, ShaoYing Ke, ShaoZe Lin, LiangJuan Chen, Zhishan Zhang, Tao Zhang

**Affiliations:** ^1^ Department of Clinical Laboratory Quanzhou First Hospital Affiliated to Fujian Medical University China; ^2^ Department of Clinical Laboratory The Hospital of Nanan City China; ^3^ Department of Clinical laboratory Yongchun Hospital of Traditional Chinese Medicine China; ^4^ Department of Immunology School of Basic Medical Sciences Fujian Medical University Fuzhou China

**Keywords:** liver cancer, matrix metalloproteinase‐9, prognosis, small ubiquitin‐like modifier, small ubiquitin‐like modifier 2, vascular endothelial growth factor

## Abstract

This study aimed to evaluate the prognostic value and biological function of small ubiquitin‐like modifier 2 (*SUMO2*) in hepatocellular carcinoma (HCC). *SUMO2* expression in HCC tissues was markedly higher than that in normal liver tissues, and patients with high *SUMO2* expression had significantly shorter median overall survival than those with low *SUMO2* expression. Furthermore, *SUMO2* expression was closely correlated with lymph node metastasis and vascular invasion and was a predictor of poor prognosis. The knockdown of *SUMO2* in two HCC cell lines (SMMC‐7721 and Bel‐7404) dramatically suppressed their proliferation, migration and invasion. Western blot analysis showed that the downregulation of SUMO2 significantly reduced the expression of Ki‐67, matrix metalloproteinase‐9 (MMP‐9) and vascular endothelial growth factor (VEGF) in SMMC‐7721 and Bel‐7404 cells. Similarly, quantitative reverse transcription–PCR revealed consistently decreased expression of *MMP‐9* and *VEGF*. Our data suggest that SUMO2 promotes proliferation, migration and invasion of HCC cells via mechanisms involving MMP‐9 and VEGF. Therefore, SUMO2 may be a prognostic factor and a promising therapeutic target for patients with HCC.

## Graphical abstract

We observed that the overexpression of small ubiquitin‐like modifier 2 (*SUMO2*) in hepatocellular carcinoma (HCC) tissues is associated with poor prognosis in patients with HCC. Silencing of SUMO2 in HCC cell lines reduced the expression of both vascular endothelial growth factor (VEGF) and matrix metalloproteinase‐9 (MMP‐9). SUMO2 promoted the tumorigenic phenotypes of HCC cells through mechanisms involving MMP‐9 and VEGF. Therefore, SUMO2 may serve as a prognostic marker and a promising therapeutic target for patients with HCC.

**Abbreviations**
AUC: area under the curve
CCK‐8: cell counting kit‐8
DMEM: Dulbecco's modified Eagle's medium
ECM: extracellular matrix
EMT: epithelial–mesenchymal transformation
GAPDH: glyceraldehyde‐3‐phosphate
GEO: Gene Expression Omnibus
HCC: hepatocellular carcinoma
LKB1: liver kinase B1
MMP‐9: matrix metalloproteinase‐9
NC: nonspecific scrambled siRNA
PD‐L1: programmed cell death ligand 1
qRT‐PCR: quantitative reverse transcription–PCR
ROC: receiver operating characteristic
SENP2: SUMO‐specific protease 2
siRNA: small interfering RNA
SIRT1: silent information regulator 1
siSUMO2: SUMO2 siRNA
SUMO: small ubiquitin‐like modifier
TCGA: The Cancer Genome Atlas
VEGF: vascular endothelial growth factor

Liver cancer ranks sixth in global cancer incidence and second in tumour‐related mortality. More than half of the new liver cancer cases and deaths occur in China, posing a serious public health challenge. Hepatocellular carcinoma (HCC) accounts for approximately 90% of all primary liver cancer cases [1, 2]. Owing to the difficulty of early diagnosis, rapid disease progression and lack of targeted drugs, patients with HCC have a poor prognosis and low 5‐year relative survival rates [3]. Therefore, the key to liver cancer control and prevention is early detection, since that would provide a significant opportunity for improving the prognosis in patients with this disease [4, 5, 6]. With the emergence of precision medicine, identification of molecular biomarkers and drug targets have become the focus of cancer research [7].

Small ubiquitin‐like modifier (SUMO) is a protein with a molecular structure that is similar to that of ubiquitin. The amino acid sequence and surface charge distribution in SUMO are different from those in ubiquitin; hence, its function is different [8]. SUMO protein was first identified in 1996. There are four SUMO subtypes in mammals: SUMO1, SUMO2, SUMO3 and SUMO4. SUMO1–3 are expressed in most tissues, whereas SUMO4 is primarily expressed in the kidney and immune system [9, 10]. The various SUMO protein subtypes play different roles. SUMO1 mainly modifies proteins that play role in cell physiology, whereas SUMO2 and SUMO3 mainly modify stress‐related proteins [11]. SUMOylation is a reversible post‐translational modification that is characterised by the covalent binding of SUMO to the target protein. SUMO attachment is catalysed by the sequential action of E1 (SAE1/SAE2), E2 (ubiquitin‐binding enzyme 9) and E3 enzymes that control modification selectivity and reaction rates in a manner similar to that during ubiquitination process [12].

SUMO modification is a crucial molecular regulatory mechanism in eukaryotic cells. It is involved in DNA damage repair, immune response, carcinogenesis, cell cycle progression and apoptosis. SUMO modification disorders are associated with several diseases, particularly cancer. For example, in leukaemia, suberoylanilide hydroxamic acid, an inhibitor of histone deacetylase, downregulates the stability of chromobox protein homolog 2 through SUMO2/3 pathway, resulting in impaired cell proliferation [13]. In the presence of latent membrane protein 1 (LMP1), the main oncoprotein of Epstein–Barr virus, the SUMOylation process in lymphoma tissues was upregulated. LMP1‐mediated cell SUMOylation disorder contributes to tumorigenesis [14]. Smad nuclear‐interacting protein 1 (SNIP1) is a transcriptional repressor of the transforming growth factor beta (TGF‐β) and nuclear factor kappa‐light‐chain‐enhancer of activated B‐cell signalling pathways, and SUMOylation of SNIP1 enhances TGF‐β‐regulated cell migration and invasion [15]. SUMOylation is necessary for the activation of hypoxia‐dependent Gli protein and affects the chemosensitivity of hepatoma cells [16]. In cells treated with mitochondrial stressors, mitofusins are conjugated to SUMO2. SUMO2 modifies mitofusins 1/2, promoting mitochondrial fusion in the perinuclear region [17].

As a prelude to this study, bioinformatic analysis of data extracted from The Cancer Genome Atlas (TCGA) and Gene Expression Omnibus (GEO) databases was performed. It was revealed that the overall survival rate in patients with high *SUMO2* mRNA expression in liver cancer tissues relative to adjacent tissues was lower than that in patients with nonelevated *SUMO2* levels. To further confirm these findings, paraffin‐embedded liver tumour tissues and adjacent tissues were collected to examine the expression levels of SUMO2 protein and analyse their correlations with the patient clinicopathological features. These preliminary studies showed that SUMO2 was upregulated in liver cancer tissues and that its high expression level was associated with poor prognosis.

Therefore, we hypothesised that SUMO2 plays a role in promoting the development of liver cancer. To further explore the influence of SUMO2 on the biological behaviour of liver cancer cells, we constructed *SUMO2*‐silenced cells and analysed the effects of *SUMO2* downregulation on cell proliferation, migration, invasion and related mechanisms.

## Materials and methods

### Patients and samples

Seventy paraffin‐embedded HCC and paired normal liver tissue samples were obtained from Quanzhou First Hospital Affiliated to Fujian Medical University, Quanzhou, China. These patients underwent surgery between 2012 and 2013 and underwent no radiotherapy and/or chemotherapy, interventional therapy, immunotherapy or traditional Chinese medicine treatment before surgery. They were followed up every 3 months from the date of surgery until January 2019; follow‐up was mainly conducted through telephone calls and the Social Security Death Index. Clinical data, including age, sex, tumour histological grade, tumour size, lymph node metastasis, vascular invasion and T stage, were obtained from the detailed electronic medical record system. The experiments were undertaken with the understanding and written consent of each subject. The study methodologies conformed to the standards set by the Declaration of Helsinki and was approved by the Ethics Committee of Quanzhou First Hospital (Approval Number: 2019143).

### Immunohistochemistry

Immunohistochemistry was performed to detect SUMO2 expression in HCC and adjacent tissues. Briefly, paraffin‐embedded HCC and paired normal liver tissue samples were sectioned into 3‐μm slices. The slices were dewaxed in xylene, hydrated in decreasing concentrations of ethanol and washed in phosphate‐buffered saline. Antigen repair was achieved by heating in citrate buffer (pH 6.0) in a pressure cooker for 2 min. Endogenous peroxide was blocked with 3% hydrogen peroxide for 10 min. The slides were incubated with a rabbit anti‐human SUMO2 polyclonal antibody (dilution 1 : 100; Abcam, Cambridge, MA, USA) overnight at 4 °C and then with biotin‐labelled secondary antibodies for 10 min at room temperature. The sections were exposed to 3,3′‐diaminobenzidine solution, and the nuclei were counterstained with haematoxylin for 20 s. Immunostaining was observed under a microscope (Olympus, Tokyo, Japan).

### Cell culture

Human HCC cell lines (SMMC‐7721 and Bel‐7404) were purchased from the Cell Bank of the Chinese Academy of Sciences (Shanghai, China) and cultured in high‐glucose Dulbecco's modified Eagle's medium (DMEM; HyClone, Logan, UT, USA) containing 10% FBS (HyClone) at 37 °C in a humidified atmosphere with 5% carbon dioxide.

### Cell transfection

Small interfering RNA (siRNA; GenePharma, Shanghai, China) was synthesised and transiently transfected into SMMC‐7721 and Bel‐7404 cells using Lipofectamine 2000 (Invitrogen, Carlsbad, CA, USA) according to the manufacturer's instructions. The sequences for *SUMO2* siRNA (*siSUMO2*) and nonspecific scrambled siRNA (NC) are shown in Table 1.

**Table 1:** siRNAs targeting specific genes.

siRNA	Sequence	
	Sense (5′–3′)	Antisense (5′–3′)
siSUMO2	GGGCAACCAAUCAAUGAAATT	UUUCAUUGAUUGGUUGCCCTT
NC	UUCUCCGAACGUGUCACCUTT	ACGUGACACGUUCGGAGAATT

### RNA isolation and quantitative reverse transcription–PCR

Total RNA was extracted from the different cell lines using TRIzol reagent (Invitrogen), and its concentration was measured using a NanoDrop One instrument (Thermo Fisher Scientific, Inc., Carlsbad, CA, USA). The RevertAid First‐Strand cDNA Synthesis Kit (Thermo Fisher Scientific, Inc.) was used for reverse transcription. Quantitative reverse transcription–PCR (qRT‐PCR) was performed using SYBR Green qPCR SuperMix (Roche, Basel, Switzerland) on an Applied Biosystems 7500 Real‐Time PCR System (Thermo Fisher Scientific, Inc.). The relative expression levels of target genes were normalised to that of glyceraldehyde‐3‐phosphate dehydrogenase (*GAPDH*) and calculated using the 2^−ΔΔCt^ method. The gene primer sequences are listed in Table 2.

**Table 2:** The primers used for RT‐qPCR.

Gene	Sequence		Product size (bp)
	Sense (5′–3′)	Antisense (5′–3′)	
SUMO2	TTTGGTGCGGACCTGGTA	TCTTAAACTGCACCACAGAACCAT	161
VEGF	TGG AGT GTG TGC CCACTG AG	TGC ATT CAC ATT TGT GCT GTA G	117
MMP‐9	TGGTCCTGGTGCTCCTGGTG	TGCCTGTCGGTGAGATTGGTTC	109
GAPDH	AGAAGGCTGGGGCTCATTTG	AGGGGCCATCCACAGTCTTC	238

### Western blot assay

Lysates from SMMC‐7721 or Bel‐7404 cells were prepared in radioimmunoprecipitation assay buffer containing 1% phenylmethylsulfonyl fluoride (Beyotime Institute of Biotechnology, Nantong, China). The lysate protein contents were separated on 8% sodium dodecyl sulfate–polyacrylamide gels and then transferred to polyvinylidene fluoride membranes (Millipore, Bedford, MA, USA). The membranes were incubated with primary antibodies against SUMO2, Ki‐67, vascular endothelial growth factor (VEGF), matrix metalloproteinase‐9 (MMP‐9), histone and GAPDH overnight at 4 °C. The membranes were then exposed to the corresponding horseradish peroxidase‐conjugated secondary antibodies for 1 h at room temperature. Finally, the antibody‐bound proteins were visualised using the ChemiDoc Touch Imaging System (Bio‑Rad, Hercules, CA, USA).

### Cell proliferation assay

Following transfection and incubation for 36 h, SMMC‐7721 and Bel‐7404 cells were seeded at a density of 3 × 10^3^ cells per well suspended in 100 µL of complete medium in a 96‐well plate. The cell counting kit‐8 (CCK‐8; Dojindo, Japan) was used according to the manufacturer's instructions, and optical density values at 450 nm were obtained at 0, 12, 24, 48 and 72 h using a BioTek Epoch Microplate Reader (BioTek, Winooski, VT, USA).

### Plate colony formation assay

SMMC‐7721 and Bel‐7404 cells were seeded into six‐well plates at a density of 3000 cells per well and cultured for 2 weeks. The cells were then fixed in 4% paraformaldehyde for 30 min and stained with 0.1% crystal violet for 15 min at room temperature. Finally, the clones were photographed and counted to assess cell proliferation.

### *In vitro* cell invasion assay

Cell invasion assays were performed using Transwell chambers with 8‐μm pore filters (Corning, New York, NY, USA). SMMC‐7721 and Bel‐7404 cells were seeded in six‐well plates and transfected with siSUMO2 or NC and incubated for 36 h. The cells were then seeded at a density of 5 × 10^4^ cells per well in 200 μL of serum‐free DMEM in the upper chamber; the bottom chamber contained 600 μL of DMEM with 10% FBS as a chemoattractant. After a 24‐h incubation, cells were fixed with methanol and stained with 0.1% crystal violet. Five random fields were photographed at ×200 magnification using a digital microscopic imaging system (Leica, Bensheim, Germany), and the cells within these fields were counted.

### Wound‐healing assay

The two HCC cell lines (control, siSUMO2 or NC) were seeded on six‐well plates and allowed to reach 80% confluency. A 200‐μL sterile pipette tip was used to generate the wounds (three scratches per well); the wells were then rinsed with phosphate‐buffered saline to remove floating cells. Representative images of cells migrating into the wounded areas were taken using a light microscope at 0, 24 and 48 h postscratching. imagej software (NIH, Bethesda, MD, USA) was used to process the images, and cell migration was evaluated by comparing the changes in gap widths between the two time points.

### Statistical analyses

The Statistical Package for the Social Sciences (spss) statistical software (version 17.0; SPSS Inc., Chicago, IL, USA) was used for data analysis. The chi‐squared or Fisher's exact test was used to determine the association between SUMO2 expression in liver cancer tissue samples and the patient clinicopathological features. Receiver operating characteristic (ROC) curves were used to detect the diagnostic significance of SUMO2. The overall survival rates were analysed using the Kaplan–Meier method and compared using the log‐rank test. Multivariate Cox regression models were used to analyse the effect of SUMO2 on patient survival and prognosis. The *in vitro* experiments were each performed three times independently; data are expressed as the mean ± standard deviation. One‐way analysis of variance was used to compare between different experimental groups, and a *P* < 0.05 was considered statistically significant.

## Results

### Small ubiquitin‐like modifier 2 is a potential biomarker for liver cancer

SUMO2 is rarely studied in tumours, and its specific role remains unclear. We reviewed public databases to mine existing data on the *SUMO2* gene in liver cancer. *SUMO2* mRNA expression levels in 421 patients (371 liver tumour tissues and 50 adjacent tissue samples) were obtained from TCGA database, whereas those from another 167 patients (115 liver tumour tissues and 52 adjacent tissue samples) were obtained from the GEO database. Our analysis revealed that *SUMO2* mRNA expression levels in liver cancer tissues were significantly higher than those in adjacent tissues (Fig. 1A,B). Meanwhile, the Kaplan–Meier analysis of 364 patients with liver cancer (www.kmplot.com; public database website) showed that the total survival time in patients with high level of *SUMO2* expression was significantly shorter than that in patients with low *SUMO2* expression level (Fig. 1C). Using public databases, we preliminarily confirmed that the expression status of *SUMO2* in liver cancer was consequential to the clinical prognosis of patients with this disease.

**Fig. 1:** SUMO2 is a potential biomarker for liver cancer. (A, B) *SUMO2* mRNA expression levels in liver cancer tissues from TCGA (normal tissue, *n* = 50; primary tumour tissue, *n* = 371) and GEO databases (adjacent nontumour tissue, *n* = 52; primary tumour tissue, *n* = 115) were significantly higher than those in respective adjacent tissues (**P < 0.001 vs normal tissue, Student's *t*‐test; the error bars indicate SD). (C) Kaplan–Meier curves of overall survival in 364 patients with HCC in the KM‐Plotter public database according to *SUMO2* expression (*P* = 0.033, Kaplan–Meier curves and log‐rank test). FC, fold change; HR, hazard ratio.

### SUMO2 protein is highly expressed in liver cancer tissues and associated with a poor prognosis

Among the 70 patients with primary liver cancer, 60 (85.7%) and 10 (14.3%) were men and women, respectively. The median age was 48 (range, 26–73) years. Thirty‐two (45.7%) patients were aged < 48 years, while 38 (54.3%) patients were aged ≥ 48 years. According to the Union of International Cancer Control classification system, 25 (35.7%) tumours were well‐differentiated, while 45 (64.3%) tumours were moderately or poorly differentiated. Thirty‐four (48.6%) patients had a maximum tumour diameter of < 7.5 cm, while 36 (51.4%) patients had a maximum tumour diameter of ≥ 7.5 cm. Thirty‐six patients (51.4%) had no lymph node metastasis, while 34 (48.6%) patients had lymph node metastasis. Thirty patients (42.9%) had no vascular invasion, while 40 (57.1%) patients had vascular invasion. According to the eighth edition of the American Joint Committee on Cancer Staging System, 30 (42.9%) and 40 (57.1%) patients had stage T1 or T2 and stage T3 or T4 disease, respectively. All patients were followed up from the date of surgery, and 50 (71.4%) patients died during follow‐up. The median survival time was 29.5 (range, 2–79) months (Table 3).

**Table 3:** Patients' characteristics.

Variable	Cases	
	(*N* = 70)	
	*N*	%
Gender		
Female	10	14.3
Male	60	85.7
Age		
< 48	32	45.7
≥ 48	38	54.3
Histologic grade		
Well differentiated	25	35.7
Moderately/poorly differentiated	45	64.3
Tumour size		
< 7.5 cm	34	48.6
≥ 7.5 cm	36	51.4
Lymph node metastasis		
No	36	51.4
Yes	34	48.6
Vascular invasion		
No	30	42.9
Yes	40	57.1
T stage		
T1 + T2	30	42.9
T3 + T4	40	57.1
Survival		
Alive	20	28.6
Dead	50	71.4

SUMO2 protein, which is mainly located in the nucleus, was highly expressed in 45 patients with HCC; hence, the expression rate was 64.3% (45/70). However, only 14 of the paired paracancerous normal tissues showed high expression of SUMO2 [expression rate, 20.0% (14/70)]; the difference in SUMO2 expression between the two tissue types was statistically significant (*P* = 0.026; Table 4 and Fig. 2A). These data were consistent with the results of our previous database analysis and indicated that SUMO2 is valuable for predicting the prognosis of patients with liver cancer.

**Table 4:** Expression of SUMO2 protein in paired normal tissues and HCC tissues

Tissues sample	*N*	SUMO2 expression		*P* value
		Low expression (%)	High expression (%)	
Normal tissues	70	56 (80.0)	14 (20.0)	0.026*
Tumour tissues	70	25 (35.7)	45 (64.3)	

* Statistically significant (*P* < 0.05).

**Fig. 2:** SUMO2 is highly expressed in liver cancer tissues and associated with a poor prognosis. (A) Representative images of SUMO2 staining in liver cancer and paired paracancerous tissues: (i) high SUMO2 expression in liver cancer tissues, (ii) low SUMO2 expression in liver cancer tissues, (iii) high SUMO2 expression in paracancerous tissues and (iv) low SUMO2 expression in paracancerous tissues. Scale bar = 100 µm. (B) Kaplan–Meier curves of overall survival in 70 patients with HCC according to SUMO2 expression (*P* < 0.001, Kaplan–Meier curves and log‐rank test). HR, hazard ratio; MST, median survival time.

We performed the Kaplan–Meier analysis to further assess whether SUMO2 expression was associated with overall survival in 70 patients with HCC. The overall survival in patients with high SUMO2 expression was shorter than that in patients with low SUMO2 expression (23.0 vs 61.0 months, respectively; *P* < 0.001), indicating that the high expression level of SUMO2 protein is a predictor of poor prognosis in patients with HCC (Fig. 2B). Next, we used a multivariate Cox regression model that included age, sex, degree of differentiation, tumour size, T stage, the presence lymph node metastasis and vascular invasion, and other clinicopathological features as variables to examine whether SUMO2 protein expression influences the prognosis of patients with HCC. This analysis revealed that lymph node metastasis, vascular invasion and SUMO2 protein expression status were independent prognostic factors (Table 5). Finally, the chi‐squared or Fisher's exact test was used to analyse the correlation between SUMO2 expression and the clinicopathological features in 70 patients with HCC. Variables included age, sex, degree of differentiation, tumour size, T stage and the presence of lymph node metastasis and vascular invasion. High expression of SUMO2 protein was found to be closely associated with lymph node metastasis (85.3%) and vascular invasion (87.5%), with a high mortality rate (82.0%), but was not significantly correlated with other clinicopathological features (Table 6). These results strongly suggest that SUMO2 protein may be an independent prognostic factor for patients with HCC.

**Table 5:** Multivariate Cox regression analyses for overall survival in HCC patients.

Characteristics	Multivariate analysis	
	HR (95% CI)	*P* value
Gender		
Female	1.00	0.846
Male	0.92 (0.38–2.21)	
Age		
< 48	1.00	0.081
≥ 48	1.69 (0.94–3.01)	
Histologic grade		
Well differentiated	1.00	0.146
Moderately/poorly differentiated	1.60 (0.85–3.00)	
Tumour size		
< 7.5 cm	1.00	0.200
≥ 7.5 cm	1.57 (0.79–3.11)	
Lymph node metastasis		
No	1.00	0.015*
Yes	2.12 (1.16–3.89)	
Vascular invasion		
No	1.00	0.021*
Yes	2.24 (1.13–4.47)	
T stage		
T1 + T2	1.00	0.350
T3 + T4	0.70 (0.34–1.47)	
SUMO2 expression		
Low expression	1.00	0.037*
High expression	2.35 (1.05–5.25)	

* Statistically significant (*P* < 0.05).

**Table 6:** Association between SUMO2 expression and clinicopathological characteristics in HCC.

Characteristics	SUMO2 expression		*P* value
	Low expression (%)	High expression (%)	
Gender			
Female	3 (30.0)	7 (70.0)	0.686
Male	22 (36.7)	38 (53.7)	
Age			
< 48	14 (43.7)	18 (52.3)	0.198
≥ 48	11 (28.9)	27 (71.9)	
Histologic grade			
Well differentiated	7 (28.0)	18 (72.0)	0.315
Moderately/poorly differentiated	18 (40.0)	27 (60.0)	
Tumour size			
< 7.5 cm	10 (29.4)	24 (70.6)	0.285
≥ 7.5 cm	15 (41.7)	21 (58.3)	
Lymph node metastasis			
No	20 (55.6)	16 (44.4)	< 0.001*
Yes	5 (14.7)	29 (85.3)	
Vascular invasion			
No	20 (66.7)	10 (33.3)	< 0.001*
Yes	5 (12.5)	35 (87.5)	
T stage			
T1 + T2	10 (33.3)	20 (66.7)	0.719
T3 + T4	15 (37.5)	25 (62.5)	
Survival			
Alive	16 (80.0)	4 (20.0)	< 0.001*
Dead	9 (18.0)	41 (82.0)	

* Statistically significant (*P* < 0.05).

### Evaluating the prognostic value of SUMO2 in liver cancer

The abovementioned results revealed a significant difference in the expression of SUMO2 protein between liver cancer tissues and paired adjacent normal tissues. High SUMO2 expression level was closely associated with lymph node metastasis, vascular invasion and a high mortality rate. Next, we examined whether ROC analysis can be utilised for diagnosing liver cancer. We found that the expression of SUMO2 protein in cancer tissues was of moderate diagnostic value, albeit with statistical significance. The diagnostic value of SUMO2 overexpression was the highest in terms of survival [area under the curve (AUC): 0.810], with a sensitivity of 82.00% and a specificity of 80.00% (Table 7 and Fig. 3A). The diagnostic values of lymph node metastasis and vascular invasion were also high (AUC: 0.704 and 0.771, respectively), with sensitivities of 85.3 and 87.5% and specificities of 55.56 and 66.67%, respectively (Fig. 3B,C). The diagnostic value of SUMO2 overexpression in terms of other diseases was low and not significant.

**Table 7:** ROC curve evaluated the diagnostic value of SUMO2 in HCC.

Characteristics	SUMO2 expression	AUC	95% CI	Sensitivity (%)	Specificity (%)	*P*
Survival	Tumor tissues	0.810	0.691–0.929	82.00	80.00	< 0.001*
	Normal tissues	0.570	0.427–0.713	24.00	90.00	0.363
Lymph node metastasis	Tumor tissues	0.704	0.580–0.828	85.30	55.56	< 0.001*
	Normal tissues	0.592	0.457–0.726	29.40	88.89	0.188
Vascular invasion	Tumor tissues	0.771	0.653–0.889	87.50	66.67	< 0.001*
	Normal tissues	0.558	0.423–0.694	25.00	86.67	0.406

* Statistically significant (*P* < 0.05).

**Fig. 3:** ROC analysis evaluating the prognostic value of SUMO2 in liver cancer. (A) Survival status, (B) lymph node metastasis and (C) vascular invasion. *n* = 70.

### SUMO2 downregulation inhibits liver cancer cell proliferation

We used siRNA to knockdown *SUMO2* expression in the liver cancer cell lines SMMC‐7721 and Bel‐7404. qRT‐PCR confirmed that *SUMO2* gene expression levels were reduced by > 75% following transfection with siSUMO2. Western blotting also confirmed the downregulation of SUMO2 protein (Fig. 4A,B). To evaluate the effect of *SUMO2* downregulation on the growth and proliferation of SMMC‐7721 and Bel‐7404 cells, we used the CCK‐8 assay and plate cloning experiments to evaluate cellular proliferation and clone formation ability. The CCK‐8 assay showed that the proliferation of siSUMO2‐transfected cells was significantly lower after 24 h compared with that in the NC and control groups (*P* < 0.05). By 72 h, the gap in proliferation between the siSUMO2 and NC or control groups had increased significantly (*P* < 0.001; Fig. 4C). Moreover, the cloning ability of SMMC‐7721 and Bel‐7404 cells was significantly reduced after siSUMO2 transfection (*P* < 0.001; Fig. 4D,E). As shown in Fig. 4F,G, the expression of Ki‐67 (a nuclear antigen that is expressed during the late stages of the cell cycle and is an indicator of proliferation) was also significantly reduced in SMMC‐7721 and Bel‐7404 cells (*P* < 0.001). These data indicated that SUMO2 played an important role in the proliferation and clone formation of SMMC‐7721 and Bel‐7404 liver cancer cells.

**Fig. 4:** The downregulation of SUMO2 inhibits liver cancer cell proliferation. (A, B) SUMO2 expression in siSUMO2‐transfected SMMC‐7721 and Bel‐7404 cells. (C) Cell proliferation measured using Cell Counting Kit‐8 assays. (D, E) Cell clone formation assessed using plate cloning experiments. (F, G) Ki‐67 expression in SMMC‐7721 and Bel‐7404 cells. (*P < 0.05 or **P < 0.01 vs the Con or NC groups, one‐way analysis of variance; the error bars indicate SD, *N* = 3, scale bar = 100 µm). Con, control; NC, nonspecific scrambled RNA; OD, optical density.

### Downregulation of SUMO2 inhibits the migration and invasion of liver cancer cells

Cell migration is not only a physiological component of cell growth and development, but also associated with tumour growth and metastasis. Therefore, we investigated whether *SUMO2* knockdown can affect the migration potential of liver cancer cells via scratch experiments. The denuded areas of plated control, NC and siSUMO2 cells were photographed at 0 and 24 h, and the differences in the widths of the gaps were calculated using imagej software. As shown in Fig. 5A,B, there was no significant difference in gap closure between the control and NC‐transfected SMMC‐7721 cells at 24 and 48 h (*P* > 0.05). However, the differences in the migration and total areas of the siSUMO2‐transfected SMMC‐7721 and Bel‐7404 cells were significantly greater than those of the control cells (*P* < 0.001). These data suggest that *SUMO2* downregulation significantly inhibits cell migration.

**Fig. 5:** The downregulation of SUMO2 inhibits liver cancer cell migration and invasion. (A, B) Cell migration in SMMC‐7721 and Bel‐7404 cells measured using a wound‐healing assay. (C, D) Cell invasion in SMMC‐7721 and Bel‐7404 cells measured using a Transwell assay. (E–G) VEGF and MMP‐9 expression in SMMC‐7721 and Bel‐7404 cells. (**P < 0.01 vs the Con or NC groups, one‐way analysis of variance; the error bars indicate SD, *N* = 3, scale bar = 100 µm). Con, control; NC, nonspecific scrambled RNA.

Transwell chambers coated with Matrigel were used to simulate the extracellular matrix (ECM) of cells in the body, and liver cancer cells that traversed the Matrigel to the lower chamber of the Transwell were enumerated. Cells transfected with siSUMO2 were significantly less abundant in the bottom chamber than their control and NC‐transfected counterparts (*P* < 0.001; Fig. 5C,D). These findings indicate that *SUMO2* knockdown can inhibit the invasive potential of liver cancer cells.

One reason for the poor efficacy of therapeutic interventions against HCC is that the tumour cells exhibit invasive and metastatic behaviours at an early stage; this is usually accompanied by the formation of tumour neovascularisation. MMP‐9 is the most common matrix metalloproteinase in the MMP family; it efficiently degrades the ECM and is believed to play an important role in tumour invasion and metastasis. VEGF is the strongest angiogenic factor in the body and is closely related to distant metastasis and tumour angiogenesis. Our analysis of clinical samples showed that the high expression of *SUMO2* was closely related to lymph node metastasis and vascular invasion. Therefore, we further investigated whether *SUMO2* knockdown affected the expression of *VEGF* and *MMP‐9* via qRT‐PCR. The expression levels of these genes in SMMC‐7721 and Bel‐7404 liver cancer cells transfected with siSUMO2 were significantly reduced compared to those in control cells (*P* < 0.001; Fig. 5E). Moreover, VEGF and MMP‐9 protein levels in both cell lines transfected with siSUMO2 were also significantly reduced (*P* < 0.001; Fig. 5F,G). Taken together, knocking down *SUMO2* expression led to the attenuation of liver cancer cell migration and invasion; this in turn appeared to be associated with the decreased expression of *VEGF* and *MMP‐9*.

## Discussion

SUMO proteins belong to a small family of protein modifiers, namely ubiquitin‐like proteins, that are conjugated to target proteins following a series of reactions catalysed by the E1‐activating enzyme, E2‐conjugating enzyme and E3 ligase [18].SUMO proteins can modify one or more lysine residues of the target protein and form multiple SUMO protein chains on the substrate molecule. SUMOylation modifies protein–protein interactions, thereby mediating the positioning and functional regulation of the target protein [19]. SUMO modification‐related disorders play an important role in the pathogenesis of several cancers, especially those associated with inflammation, as is the case with liver cancer [20, 21].

SUMO‐specific protease 2 (SENP2) is one of the most common proteases known to reverse SUMO modification. Its expression is low in HCC, and its overexpression inhibits the growth and colony formation of HCC cells. As such, SENP2 is considered a tumour suppressor; moreover, it also regulates β‐catenin [22, 23]. Ubiquitin‐binding enzyme 9 is an essential SUMO‐modified enzyme that is highly expressed in liver cancer [24]. Zubiete‐Franco *et al*. [25] found that the SUMOylation of liver kinase B1 (LKB1) was enhanced in preclinical HCC mouse models and in more aggressive HCC clinical tumours. Further studies showed that SUMO2 modifies endogenous LKB1, the extent of which is higher in fast‐growing tumours. Therefore, SUMO modification is thought to regulate the localisation of LKB1 and its carcinogenic activity in liver cancer. Liu *et al*. [26] found that SUMO2/3 and P65 levels were closely correlated in liver cancer and that their interaction was promoted by tumour necrosis factor‐α. This stabilisation of cytoplasmic P65 may represent a novel mechanism for the development of HCC as a result of chronic hepatitis. Therefore, it is hypothesised that SUMO modification and the SUMO protein itself play important roles in liver carcinogenesis.

Our screening for the differential expression of *SUMO2* in liver cancer vs adjacent tissues using TCGA and GEO databases revealed that *SUMO2* was highly expressed in the former and that the prognosis in patients with high *SUMO2* expression was worse than that in patients with low *SUMO2* expression. To further investigate this, 70 clinical samples comprising cancer and paracancerous tissues were analysed for their SUMO2 protein expression levels, wherein we found that SUMO2 protein was highly expressed in 45 of the 70 HCC tissue specimens where it was mainly localised in the nucleus. Statistical analysis of the clinicopathological features of these 70 patients as related to SUMO2 protein expression showed that elevated SUMO2 was closely associated with high mortality, lymph node metastasis and vascular invasion (i.e. higher SUMO2 protein levels in cancer tissues were positively correlated with proliferation, migration and invasion). This contrasts with the findings of Liu *et al*. [26], who found that SUMO2/3 was downregulated in hepatitis B virus‐infected liver cancer tissues. This may be related to differences between samples. Moreover, SUMO2 and SUMO3 may have different functions. Owing to their sequence homology, these two proteins were once considered indistinguishable, which is why they were referred to as SUMO2/3 [27]. However, a more recent study has found that the two isoenzymes have different regulatory mechanisms, and their transcription is related to the differential regulation of Sp1‐dependent oxidative stress [28]. Based on our results, SUMO2 can be used as an independent prognostic factor for patients with liver cancer and can positively regulate the migration and invasion of HCC cells. We demonstrated the role of SUMO2 as a key cancer‐promoting factor using siRNA technology to knock down the expression of the target gene in liver cancer cells, which significantly inhibited their proliferation, migration and invasion.

Cancer cells undergo numerous characteristic changes during tumour progression. These include the ability to promote growth or inhibit growth signals independently of exogenous stimuli, invade surrounding tissues, metastasise to distant locations, trigger angiogenic responses and evade mechanisms that limit cell proliferation, such as apoptosis and replicative senescence. These characteristics reflect changes in signalling pathways that control cell proliferation, migration and survival in normal cells [29]. Cell proliferation is important for the development of tumour malignant potential. In this study, we constructed liver cancer cells with silenced SUMO2 protein and found their proliferation and colony‐forming abilities to be significantly reduced, indicating the importance of SUMO2 in these behaviours.

Ki‐67, which is not expressed in resting cells, but is ubiquitous in all proliferating normal and tumour cells, is an excellent marker for determining the growth potential of a given cell population. The expression of Ki‐67 is closely related to the proliferation and growth of tumour cells and is widely used as a proliferation marker in routine pathological studies [30, 31, 32]. In our study, we observed that the downregulation of SUMO2 significantly reduces Ki‐67 staining in liver cancer cells, further indicating that the high expression of SUMO2 protein promotes the occurrence and development of liver cancer. Tumour metastasis involves the migration and seeding of cancer cells at secondary sites and is the cause of most cancer‐related deaths. Therefore, the most important measure to reduce morbidity and mortality is the prevention or eradication of tumour metastases [33].

In our study, siSUMO2‐transfected liver cancer cells had a slower *in vitro* wound‐healing rate in scratch assays and diminished invasion through Matrigel. This was consistent with our data from clinical sample analyses showing that high SUMO2 expression in liver cancer was closely associated with tumour invasion and metastasis. Epithelial–mesenchymal transformation (EMT) is the process by which epithelial cells acquire mesenchymal characteristics; in cancer, EMT is associated with tumour growth, invasion, metastasis and chemoresistance [34]. Silent information regulator 1 (SIRT1) plays an important role in inhibiting ovarian cancer tumorigenesis and metastasis by preventing EMT *in vivo* and *in vitro* [35].

A previous study reported that the SUMO E3 ligase protein inhibitor of activated signal transducer and activator of transcription 4 was induced by hypoxia, which prevents Sp1 from binding to the SIRT1 promoter in cancer cells, thereby promoting tumour development [36]. VEGF, which is a key mediator of angiogenesis in cancer, is both a vascular growth and permeability factor and is upregulated by oncogenes, various growth factors and hypoxia, thus promoting tumour metastasis [37, 38]. Many immunosuppressive mechanisms involved in the recurrence of HCC are regulated by VEGF and/or immune checkpoints, such as programmed cell death ligand 1 (PD‐L1). Studies have shown that the PD‐L1 inhibitor atezolizumab and VEGF inhibitor bevacizumab can significantly improve the overall survival, progression‐free survival and overall response rates in patients with unresectable HCC. The combined blockade of PD‐L1/VEGF may effectively reduce the recurrence of HCC [39]. Moreover, tumour cells that metastasise to other organs must locally degrade the ECM components. The MMP family comprises key enzymes facilitating this process, and the degradation of the ECM by MMPs enhances tumour invasion [40]. The most widely studied metalloproteinase, MMP‐9, can cleave many ECM proteins and promote ECM remodelling. A large number of studies have found that MMP‐9 promotes cancer‐related phenotypes, including invasion, metastasis and angiogenesis [41], and the overexpression of MMP‐9 promotes cancer metastasis. Lu *et al*. [42] found that the long noncoding RNA FLJ33360 was upregulated in liver cancer and that it accelerated the metastasis of HCC by targeting the miRNA‐140/MMP‐9 axis. In this study, we found that silencing SUMO2 reduced the expression of both VEGF and MMP‐9 in liver cancer cells.

Our experiments showed that SUMO2 plays an important role in the occurrence and development of liver cancer. The post‐translational modification of LKB1 may be related to HCC [43]. A study has found that the SUMO2 modification of LKB1 at Lys178 mediated the nucleocytoplasmic shuttling of LKB1 and promoted the growth of liver cancer cells [25]. Therefore, it is important to clarify the specific mechanisms of downstream molecules or pathways regulated by SUMO2 to further understand the mechanism of its regulation of liver cancer pathogenesis.

In conclusion, SUMO2 is highly expressed in liver cancer tissues and associated with tumour metastasis and poor prognosis. SUMO2 upregulation enhances the tumorigenic phenotypes of liver cancer cells, such as proliferation, migration and invasion. However, the mechanism through which SUMO2 promotes the occurrence and development of HCC remains unclear, and the key proteins or signalling pathways involved need to be further characterised. This will identify more effective prognostic markers and provide new ideas for the development of targeted therapeutic drugs in clinical practice.

## Conflict of interest

The authors declare no conflict of interest.

## Author contributions

ZZ and TZ conceived and supervised the study; JC and TZ designed the experiments; JC, CC, YL, YS and XY performed the experiments; YJ, ZC, SYK, SZL and LJC analysed the data; JC and CC wrote the manuscript; and ZZ and TZ revised the manuscript.

## Data Availability

The analysed data sets generated during the study are available from the corresponding author on reasonable request.
